# Efficacy, Safety, and Prognosis of Sequential Therapy with Tamoxifen and Letrozole versus Letrozole Monotherapy for Breast Carcinoma

This article has been retracted.

**DOI:** 10.1155/2022/1979254

**Published:** 2022-04-14

**Authors:** Xinli Lu, Cheng Qian

**Affiliations:** ^1^Pharmacy Intravenous Admixture Services, the First People's Hospital of Ningyang County, Tai'an 271400, Shandong, China; ^2^Department of Thyroid and Breast Surgery, Zhuji People's Hospital of Zhejiang Province, Zhejiang 311800, China

## Abstract

**Objective:**

To explore the efficacy, safety, and patient prognosis of letrozole (LTZ) alone or in sequence with tamoxifen (TAM) for the treatment of breast carcinoma (BC).

**Methods:**

In this retrospective study, 150 patients with BC who received treatment in the First People's Hospital of Ningyang County between January 2012 and January 2017 were selected. According to different treatment methods, 99 cases receiving sequential therapy with TAM and LTZ were included in the research group, and the remaining 51 patients receiving LTZ monotherapy were selected as the control group. The efficacy, safety, survival rate, recurrence rate, and blood lipid indices (total cholesterol, TC; triglyceride, TG; high-density lipoprotein cholesterol, HDL-C; and low-density lipoprotein cholesterol, LDL-C) of the two groups were observed and compared.

**Results:**

The overall response rate of the research group was statistically higher than that of the control group, and the incidence of adverse reactions was significantly lower. No evident difference was observed in 1-, 3-, or 5-year survival rates between the two groups, while the 3-5-year recurrence rate was obviously lower, and the improvement of blood lipid indices was significantly better in the research group compared with the control group.

**Conclusion:**

LTZ alone or in sequence with TAM is effective and safe for the treatment of BC, which can significantly improve the prognosis and blood lipid indices of BC patients.

## 1. Introduction

Breast carcinoma (BC) is a genetically heterogeneous fatal disease and a common female cancer [1]. According to epidemiological data, there are approximately 2.3 million new cases of BC and 685,000 deaths worldwide [2]. With the constant optimization of BC screening methods and treatments in recent years, its recurrence rate and mortality rate have been declining, with a 5-year overall survival rate even over 90% in some countries [3]. However, once BC has metastasized, the average 5-year survival rate is as low as 22%, with certain risk of recurrence [4]. Recurrence or posttreatment complications are the main causes of morbidity and mortality in BC patients [5, 6]. Therefore, analyzing the clinical effects of treatment methods from the perspective of efficacy, safety, and patient prognosis is of great significance for reducing the mortality and recurrence rate of BC, which can also provide new clinical references for BC treatment.

This study mainly analyzes the clinical therapeutic effect of sequential therapy with tamoxifen (TAM) and letrozole (LTZ) versus LTZ monotherapy in the treatment of BC. It is shown that the tumor tissue of most BC patients is estrogen-dependent, and inhibiting estrogen stimulation of tumors can help to curb cancer progression [7]. Both TAM and LTZ are common antiestrogen drugs in clinic [8]. Among them, TAM is an antitumor drug, which is used as an estrogen receptor regulator in adjuvant endocrine therapy for hormone-dependent BC [9, 10]. LTZ, a common endocrine drug, is an aromatase inhibitor that blocks estrogen synthesis by inhibiting the final step of the estrogen biosynthesis pathway [11]. Since the effect of LTZ monotherapy is not satisfactory, it is often used in combination with other drugs or in sequence with TAM to improve the efficacy of BC treatment [8, 12]. Previous studies have shown that LTZ in sequence with TAM can increase the efficacy and safety of patients with early-stage BC to a certain extent [13]. Herein, we will analyze the effects of the two treatment methods on the clinical effect of BC patients from a more multidimensional perspective, aiming at providing a more comprehensive reference for clinical treatment of BC.

## 2. Materials and Methods

### 2.1. General Data

This is a retrospective study. A total of 150 BC patients admitted to the First People's Hospital of Ningyang County from January 2012 to January 2017 were selected and grouped according to treatment methods. Among them, 99 patients treated with sequential therapy with TAM and LTZ were included in the research group, and 51 patients treated with LTZ monotherapy were assigned to the control group. Inclusion criteria are as follows: diagnosis of BC, nonspecial invasive carcinoma, no history of contraindications to the study medication, normal cognitive and communication skills, and nonlactating and nonpregnant patients. Exclusion criteria are as follows: malignant tumor (s), other breast diseases, endocrine diseases or infectious diseases, prior treatment, and use of estrogen drugs in the past three months. This study was approved by the Ethics Committee of the First People's Hospital of Ningyang County, and all the subjects provided informed consent.

### 2.2. Treatment Methods

Patients in the control group were given LTZ (Beijing Kaishiyuan Biotechnology Co., Ltd., SC05834), per os, 2.5 mg once a day, for 5 years.

The research group was treated with LTZ sequentially following initial TAM therapy. Subjects received TAM citrate tablets (Hengyang Jinyi Biotechnology Co., Ltd., 54965-24-1) 10 mg orally twice daily for 2 years, followed by LTZ for 3 years as described above.

### 2.3. Efficacy Evaluation

Complete response (CR): all lesions disappeared for at least one month, and the remission time increased with the treatment time. Partial response (PR): the lesion basically disappeared or shrank by at least 50%, and this state was maintained for at least one month. Stable disease (SD): the lesion changed little. Progressive disease (PD): the lesion progressed with distant metastasis or lesion increase by at least 25%. The overall response rate (ORR) was the sum of CR rate and PR rate.

### 2.4. Outcome Measures

*Safety*. The incidence rates of nausea and vomiting, hyperlipidemia, thromboembolism, and muscle and joint pain were recorded in both groups, and the total incidence of adverse reactions was calculated.

*Prognosis*. The 1-year, 3-year, and 5-year survival rates as well as the 1-year, 1-3-year, and 3-5-year recurrence rates, were evaluated in both groups. The subjects were followed up every three months through telephone interviews, visits, and pathological data inquiries.

*Blood lipid indices*. Total cholesterol (TC) and triglyceride (TG), as well as high- and low-density lipoprotein cholesterol (HDL-C/LDL-C), were detected using a blood lipid analyzer (Shanghai Xinfan Biotechnology Co., Ltd., ZDSJ082).

### 2.5. Statistical Analysis

SPSS 17.0 (IBM SPSS, Madrid, Spain) and GraphPad Prism 6 (GraphPad Software, San Diego, California, USA) were used for data analysis and image rendering, respectively. Number of cases/percentages (*n*/%) was used to represent the counting data, and the comparison was performed by the Chi-square test. The measurement data were described as mean ± SEM, and the statistical methods for intergroup and intragroup comparisons were independent samples *t*-test and paired *t*-test, respectively. The significance level was set at *P* < 0.05.

## 3. Results

### 3.1. The General Data of the Two Groups Were Comparable

The research group and the control group showed no significant difference in general data such as age, average age, tumor staging, histological type, operation mode, drinking history, smoking history, and marital status (*P* < 0.05) (Table 1**)**.

### 3.2. The Efficacy of the Research Group Was Significantly Higher than That of the Control Group

The cases of CR, PR, SD, and PD in the control group were 7, 13, 17, and 14, respectively, while the corresponding cases in the research group were 30, 27, 19, and 23. The ORR of the research group was 57.57%, which was higher than that of the control group (39.22%), with statistical significance (*P* < 0.05) (Table 2**)**.

### 3.3. The Incidence of Adverse Reactions in the Research Group Was Significantly Lower than That in the Control Group

The cases of nausea and vomiting, hyperlipidemia, thromboembolism, and muscle and joint pain in the control group were 8, 6, 5, and 4, respectively, and the corresponding cases in the research group were 5, 3, 2, and 0. The total incidence of adverse reactions was 10.10% in the research group and 45.09% in the control group, with statistical significance between the two groups (*P* < 0.05) (Table 3**)**.

### 3.4. There Was No Significant Difference in Patient Prognosis between the Research Group and the Control Group

In terms of survival, the 1-year, 3-year, and 5-year survival rates of the research group were not significantly different from those of the control group (*P* > 0.05). As to recurrence, the 1-year and 1-3-year recurrence rates showed no significant difference between the two groups (*P* > 0.05). However, the 3-5-year recurrence rate was lower in the research group compared with the control group, with statistical significance (*P* < 0.05) (Table 4**)**.

### 3.5. The Blood Lipid Indices of the Research Group Were Significantly Better than Those of the Control Group after Treatment

We also compared serum lipids between the two groups, and the data showed no significant difference in lipid indices before treatment (*P* > 0.05). In the control group, the four blood lipid indices (TC, TG, HDL-C, and LDL-C) did not change significantly before and after treatment (*P* > 0.05). However, after treatment, TC, TG, and LDL-C were lower and HDL-C was higher in the research group compared with the control group, with statistically significant differences (*P* < 0.05) (Figure 1).

## 4. Discussion

BC is a common gynecological malignant tumor, seriously threatening women's physical and mental health and even life [14]. The pathogenesis of BC is complex and has not been thoroughly clarified [15]. However, most BCs are identified as estrogen-dependent tumors, and the treatment breakthrough of this disease is to inhibit the stimulation of estrogen to tumor cells [16]. The two drugs used in this study, TAM and LTZ, have varying degrees of resistance to estrogen [17]. Among them, TAM can inhibit the binding of normal progesterone, estrogen, and receptors in the body by binding to the epidermal hormone receptors of BC cells, thus preventing tumor growth [18, 19], while LTZ can restrain the growth of estrogen-dependent BC cells via inhibiting aromatase activity [20].

In this study, 99 patients treated with LTZ sequentially following initial TAM therapy were set as the research group, and 51 patients treated with LTZ monotherapy were taken as the controls. The analysis of clinical efficacy revealed a statistically higher ORR of the research group compared with the control group (57.57% *vs*. 39.22%). This suggests that the efficacy of the sequential therapy with LTZ and TAM has a significantly higher efficacy than LTZ monotherapy, which may be related to the negative impact of drug resistance on efficacy under monotherapy. It has also been pointed out that TAM resistance, the main obstacle to BC treatment, can be overcome by blocking the production of estrogen, thus improving the clinical effect [21]. With TAM sequential treatment with LTZ, LTZ as an antiestrogen drug may be beneficial to activate the pharmacological activity of TAM in patients, thus improving the ORR. In terms of safety, the two groups of patients in this study mainly had complications such as nausea and vomiting, hyperlipidemia, and thromboembolism, which were similar to some previous studies [22, 23]. In addition, this research identified a statistically lower incidence of adverse reactions in the research group compared with the control group (10.10% *vs*. 45.09%), indicating that LTZ in sequence with TAM improves patient safety. In the analysis of prognosis, no significant difference was found in the survival rate between groups, but the 3-5 year recurrence rate was significantly lower in the research group compared with the control group (11.11% *vs*. 31.37%), which suggests that the sequential treatment can reduce the recurrence risk of patients to a certain extent. In the study of Regan et al. [24], it was pointed out that sequential therapy of TAM and LTZ did not significantly improve the prognosis of BC patients compared with LTZ alone, but had a beneficial effect on the recurrence risk and treatment tolerance of patients. Finally, we analyzed the blood lipid indices and found that the blood lipid indices of the research group receiving sequential therapy with TAM and LTZ were significantly better, suggesting that the sequential treatment had some beneficial effects on improving the blood lipid of patients. Del Mastro et al. [25] also confirmed that sequential therapy with TAM and LTZ was the best standard treatment strategy for postmenopausal hormone-receptor-positive BC patients, which is similar to the results of our study.

The novelty of this study is to confirm that the sequential therapy with TAM and LTZ has a better clinical effect in the treatment of BC, as it can significantly improve the efficacy, safety, prognosis, and lipid indices of patients, which provides a more detailed clinical reference for the management of BC patients. However, there is still room for improvement in this study. First, we can increase the clinical sample size to improve the accuracy of experimental results. Second, inflammatory factors, oxidative stress, and other indicators can be detected to further supplement the effects of the two drug therapies on these indicators. Third, the analysis of risk factors affecting recurrence of BC patients can be supplemented to verify whether there is a certain correlation between medication pattern and recurrence of patients. We will conduct supplementary studies from the above perspectives in the future.

## 5. Conclusion

To sum up, either LTZ alone or in sequence with TAM for BC can not only improve the efficacy and safety of patients but also help to improve their prognosis and lipid indices, providing new insights into the mode of medication for patients with BC.

## Figures and Tables

**Figure 1:** Blood lipid indices of two groups of patients. Note: ^∗∗^*P* < 0.01.

**Table 1:** Baseline data of patients in the two groups (*n*(%), mean ± SEM).

Variables	*n*	Control group (*n* = 51)	Research group (*n* = 99)	*χ* ^2^/*t*	*P*
*Age (years)*				0.304	0.581
<65	87	28 (54.90)	59 (59.60)		
≥65	63	23 (45.10)	40 (40.40)		
Average age (years)	150	64.04 ± 6.59	63.76 ± 11.37	0.162	0.871
Course of disease (weeks)	150	10.50 ± 2.90	10.86 ± 5.10	0.466	0.642
*Tumor staging*				1.203	0.273
Stage II	50	20 (39.22)	30 (30.30)		
Stage III	100	31 (60.78)	69 (69.70)		
*Histological type*				0.061	0.806
Invasive ductal carcinoma	98	34 (66.67)	64 (64.65)		
Invasive lobular carcinoma	52	17 (33.33)	35 (35.35)		
*Operation mode*				0.132	0.716
Breast reservation radical correction	44	14 (27.45)	30 (30.30)		
Others	106	37 (72.55)	69 (69.70)		
*History of drinking*				0.942	0.332
No	98	36 (70.59)	62 (62.63)		
Yes	52	15 (29.41)	37 (37.37)		
*History of smoking*				0.135	0.713
No	97	34 (66.67)	63 (63.64)		
Yes	53	17 (33.33)	36 (36.36)		
*Marital status*				0.600	0.439
Single	35	10 (19.61)	25 (25.25)		
Married	115	41 (80.39)	74 (74.75)		

**Table 2:** Efficacy of two groups of patients (*n*(%)).

Groups	*n*	Complete response	Partial response	Stable disease	Progressive disease	Total effective rate (%)
Control group	51	7 (13.73)	13 (25.49)	17 (33.33)	14 (27.45)	20 (39.22)
Research group	99	30 (30.30)	27 (27.27)	19 (19.19)	23 (23.24)	57 (57.57)
*χ* ^2^ value	-	-	-	-	-	4.542
*P* value	-	-	-	-	-	0.033

**Table 3:** Incidence of adverse reactions in two groups (*n*(%)).

Categories	Control group (*n* = 51)	Research group (*n* = 99)	*χ* ^2^ value	*P* value
Nausea and vomiting	8 (15.69)	5 (5.05)	-	-
Hyperlipoidemia	6 (11.76)	3 (3.03)	-	-
Thromboembolism	5 (9.80)	2 (2.02)	-	-
Muscle and joint pain	4 (7.84)	0 (0.00)	-	-
Total	23 (45.09)	10 (10.10)	24.025	<0.001

**Table 4:** Prognosis of patients in two groups (*n*(%)).

Categories	Control group (*n* = 51)	Research group (*n* = 99)	*χ* ^2^ value	*P* value
1-year survival rate	47 (92.16)	94 (94.95)	0.042	0.838
3-year survival rate	44 (86.27)	85 (85.86)	0.005	0.945
5-year survival rate	37 (72.55)	79 (79.80)	1.009	0.315
1-year recurrence rate	3 (5.88)	4 (4.04)	0.257	0.612
1-3-year recurrence rate	7 (13.73)	8 (8.08)	0.275	1.192
3-5-year recurrence rate	16 (31.37)	11 (11.11)	9.362	0.002

## Data Availability

The labeled dataset used to support the findings of this study is available from the corresponding author upon request.
